The article "How Do Combustion and Non-Combustion Products Used Outdoors Affect Outdoor and Indoor Particulate Matter Levels? A Field Evaluation Near the Entrance of an Italian University Library" was published in 2020. Journal: Int J Environ Res Public Health.

# How Do Combustion and Non-Combustion Products Used Outdoors Affect Outdoor and Indoor Particulate Matter Levels? A Field Evaluation Near the Entrance of an Italian University Library

**DOI:** 10.3390/ijerph17145200

**Published:** 2020-07-18

**Authors:** Vittoria Cammalleri, Daniela Marotta, Carmela Protano, Matteo Vitali, Paolo Villari, Maria Sofia Cattaruzza, on behalf of the Smoke-free Department Working Group

**Affiliations:** Department of Public Health and Infectious Diseases, Sapienza University of Rome, 00185 Rome, Italy; vittoria.cammalleri@uniroma1.it (V.C.); daniela.marotta@uniroma1.it (D.M.); carmela.protano@uniroma1.it (C.P.); matteo.vitali@uniroma1.it (M.V.); paolo.villari@uniroma1.it (P.V.)

**Keywords:** tobacco smoking, air pollution, particulate matter, conventional cigarettes, electronic cigarettes, heat-not-burn tobacco products

## Abstract

Particulate Matter (PM) is a well-known health risk factor and pollutes both outdoor and indoor air. Using PM as an air pollution indicator, the aims were to assess outdoor and indoor air pollution due to combustion and/or non-combustion products used outdoors and to compare the PM levels emitted by different products. PM with an aerodynamic diameter ≤10, 4, 2.5 and 1 µm (PM_10_, PM_4_, PM_2.5_, PM_1_) was simultaneously measured in two areas, respectively, indoors (with smoking ban) and outdoors (where people commonly smoke) of a university library during the morning and the afternoon of two weekdays. Both combustion and non-combustion products determined a relevant worsening of outdoor air quality, with the highest PM_1_ levels achieved when a single traditional cigarette (9920 µg m^−3^), a single e-cigarette (9810 µg m^−3^) and three simultaneous traditional cigarettes (8700 µg m^−3^) were smoked. An increase of indoor PM_1_ levels was found during outdoor smoking/vaping sessions, persisting also after the end of sessions. The results highlighted the need for a revision of smoke-free laws, especially for outdoor areas, to include non-combustion products. In addition, it is essential to make society aware of the dangers of smoking outdoors by implementing health promotion interventions.

## 1. Introduction

Tobacco smoking represents one of the biggest global health hazards and a major public health issue. About seven million people worldwide die every year due to tobacco use [1]. Smoking can determine many negative effects on health through the life-course and dramatically affects the quality of life and life expectancy [2]. It is the main risk factor for the development and manifestation of cardiovascular and pulmonary diseases, including high rates of cancers, especially lung cancer. Indeed, tobacco smoke is a complex aerosol of chemical compounds bound to aerosol particles or free in the gas phase, and it composed of thousands of substances generating by incomplete combustion of tobacco during the smoking of cigarettes and other tobacco products. This smoke contains a number of toxic compounds and groups of chemicals, including carcinogenic agents such as polycyclic aromatic hydrocarbons. The chemical composition of smoke also depends on puff frequency, intensity, volume, and duration at different stages of cigarette consumption [3]. Thus, tobacco products release into the environment a great number of pollutants both during their use and when extinguished due to cigarette butts [4].

Traditionally, smoking is associated to the indoor air contamination as it dramatically increases indoor levels of air pollutants, both during and after smoking [5]. Indeed, pollutants persist in the air also when smoking products have been extinguished, representing a risk of passive smoking, also called Environmental Tobacco Smoke (ETS). This is the combination of two phenomena: Second-Hand Smoke (SHS) and Third-Hand Smoke (THS) [6]. ETS is an issue of great public health concern because it has been linked with a large number of pathologies, including cardiovascular, respiratory and neoplastic ones [7,8,9]. In addition to the worsening of indoor air quality, scientific evidence demonstrated that smoking may also be considered a source of outdoor pollution, since it produces pollutants which can contaminate outdoor air and persist for a long time [10,11,12].

Recently tobacco companies are marketing new non-combustion products (electronic cigarettes and heat-not-burn tobacco products (HTPs)) with the purpose to reduce toxic exposures and to provide harm reduction for smokers [13]. Although these products appear to emit fewer pollutants than traditional tobacco products [14], they contribute to air contamination and constitute an additional health risk [15,16,17]. The study of chemicals released during the use of e-cigs and recent HTPs have revealed to contain toxics such as carbonyls, volatile organic compounds (VOCs) and several inorganic elements, including toxic metals such as nickel, zinc and silver. However, a complete characterization of these products is still under evaluation [18]. Very recently, in Italy, the Ministry of Health reported that “it is not possible, at this stage and on the basis of the documentation provided [by the tobacco industry], to recognise the reduction of toxic substances [in HTPs] as compared to products from combustion, under the same conditions of use” [19] Thus, they represent an additional threat for passive smoking exposure

One of the main contaminants emitted by tobacco products is Particulate Matter (PM), that consists of all substances suspended in air in the form of atmospheric aerosols and, regardless of its composition, is a well-known risk factor for human health [20]. PM is categorized in different sizes according to its aerodynamic diameter. Particles especially relevant for human health are equal or smaller than 10 µm and called PM_10_ [15]. Indeed, particles, depending on their dimension, can settle on different levels of respiratory tract, reach the gas exchange regions and penetrate into the bloodstream [21,22]. Consequently, over the years, PM has been associated to several diseases, such as cardiovascular and respiratory disorders [23,24]. Besides, PM is also a major environmental risk factor for the development of some neurodegenerative diseases [25]. Exposure to PM during pregnancy has been linked with negative birth outcomes [26]. In addition, outdoors PM has been classified as Group 1 carcinogen by the International Agency for Research on Cancer (IARC) [20]. PM can pollute both outdoor and indoor air and can derive from natural (fires, volcanic eruptions, etc.) and human (vehicular traffic, heating systems, tobacco smoke) sources [22]. In particular, scientific evidences demonstrated that smoking is one of the major sources of indoor PM both from traditional tobacco products [27] or electronic devices [28,29].

In order to protect human health of smokers and non-smokers from ETS exposure in enclosed environments, many countries introduced smoking bans in indoor public places; also, several countries introduced smoking ban in some outdoor public places, such as hospitals, parks, schools [30]. In particular, the Smoke-free Environment Act 2000 made several outdoor public places smoke free [31]. However, smoking is still allowed in outdoor public areas such as streets, parks, universities, etc., despite the laws and the evidences of its contribution to outdoor pollution and the possibility of ETS exposure also outdoor [10,11,12,32].

Besides, new possible threats for ETS exposure emerge from the use of electronic cigarettes and heat-not-burn devices. Indeed, while indoor passive smoking risk connected to these products needs additional evidence [17], no studies (to our knowledge) evaluated outdoor air contamination during their use.

Using PM as a global indicator of air pollution, the aims of the present study were: to assess outdoor air pollution due to combustion and/or non-combustion products smoked outdoor and to speculate on the potential SHS exposure of a subject standing near the smoker/s; to evaluate the contribution of smoking combustion and non-combustion products, smoked outside in the proximity of a building, on its indoor air quality and to compare the levels of PM emitted by different smoking combustion and non-combustion products.

## 2. Materials and Methods

### 2.1. Environmental Assessment of Outdoor and Indoor PM Levels

Levels of PM with an aerodynamic diameter smaller than respectively 10, 4, 2.5 and 1 µm (PM_10_, PM_4_, PM_2.5_ and PM_1_) emitted by smoking outdoor combustion products (traditional and hand-rolled cigarettes) and non-combustion products (electronic cigarettes and unheated tobacco products) were measured to assess environmental contamination. This evaluation was part of a university project for the expansion of smoke-free areas.

The PM measurements were performed in two areas, respectively, indoors and outdoors of the “Del Vecchio” library of the Department of Public Health and Infectious Diseases of Sapienza University of Rome. The indoor environment was the library’s entrance hallway located at the first floor of the Department, while the outdoor environment was the gallery on the same floor (Figure 1).

The library is located in an area without outdoor vegetation nor automobile traffic or other known sources of PM. Outdoor and indoor PM measurements took place during a morning and an afternoon of two typical weekdays.

In total, a 10-h measurement was performed; types and start/end time of each individual smoked/vaped product were registered. The smokers were university students and employees attending the library. Measurements were performed by means of two portable, laser-operated aerosol mass analyzer Dusttrak ™ II Aerosol Monitor, model 8532, 0.1–10 µm particle size range (TSI, Shoreview, MN, USA). The aerosol levels for each size fraction (PM_10_, PM_4_, PM_2.5_, PM_1_), expressed in µg m^−3^, were measured in “cumulative” mode, that is including the mass of all particles that are smaller than or equal to the defined size. The indoor aerosol was sampled directly through the entry of the instrument, positioned at about 1 m above the floor level, without using any tube, thus simulating the breathing zone of a passive, exposed, sitting subject. The outdoor aerosol was sampled through a tube placed approximately 1.5 m above floor level, connected to the second instrument, for simulating the breathing zone of a standing subject.

The indoor air exchange rate (λ) was calculated using the tracer gas technique, as previously reported [21]. Mean values of air temperature and relative humidity in indoor and outdoor environments were respectively 26.2 °C and 44.2% and 29.7 °C and 44.4%. Wind conditions were stable and low-dynamic in both the monitoring days. Meteorological parameters were measured by the use of DELTA OHM-HD 32.3 Thermal microclimate instrument (DELTA OHM Srl, PD, Italy) equipped with the probes HP3217R, AP3203, TP3275 (DELTA OHM Srl, PD, Italy) installed near the aerosol monitor indoor and outdoor. Parameters were measured in absence of direct solar irradiation. In addition, we recorded meteorological data of the Meteorological Service of the Italian Air Force headquarters.

### 2.2. Comparison of PM Levels Generated by Combustion and Non-Combustion Products

The levels of PM generated by selected combustion and non-combustion products smoked/vaped during the measuring sessions were compared. In particular, we considered six smoking/vaping sessions in which different products were smoked/vaped: one conventional cigarette (cig), one hand-rolled cigarette (RYO: Rolled Your Own), one electronic cigarette (e-cig), one iQOS^®^ (Philip Morris International), one JUUL^®^ (JUUL Labs, Inc.), one GLO^®^ (British American Tobacco). We compared the PM levels measured from about one minute before to one minute after each of the selected smoking/vaping session.

### 2.3. Statistical Analysis

The Mann–Whitney test was used to assess possible differences in median values of outdoor PM_1_ measured, respectively, before and during each of the six selected smoking/vaping sessions.

We considered just PM_1_ fraction because this fraction was the main size range (>95%) of the aerosol generated during the smoking/vaping sessions. Statistical elaboration was carried out using IBM SPSS Statistics 25 statistical software (IBM Corp., Armonk, NY, USA).

## 3. Results

### 3.1. Environmnetal Assessment of Outdoor and Indoor PM Levels

Figure 2 and Figure 3 show the levels of PM_1_ measured outdoors and indoors, respectively, during the afternoon and the morning measuring sessions.

Data reported in Figure 2a,b and Figure 3a–c show a relevant worsening of outdoor air quality during all the smoking sessions. The highest PM_1_ levels, expressed in Log_(10)_PM_1_, are reached when the following products have been smoked: three traditional cigarettes at the same time (8700 µg m^−3^), a single e-cigarette (9810 µg m^−3^) and a single traditional cigarette (9920 µg m^−3^). These values were, respectively, about 323, 446 and 451 times higher the external bottom values. Notice that the outdoor PM levels remain higher than the background level also when the cigarettes or the other products were extinguished. Figure 2c,d and Figure 3d–f) highlight also an increase of indoor PM_1_ levels in correspondence to the outdoor smoking/vaping sessions which persisted for a variable period of time even after the end of the sessions.

In both figures, the red and blue dotted lines indicate the WHO air quality guideline values for 24-h mean levels of PM_10_ and PM_2.5_ that were, respectively, 25 and 50 µg m^−3^ [33]. Since there were no specific limit values for tobacco smoke, we used WHO values for atmospheric PM levels as landmark values. As evidenced in Figure 2 and Figure 3, PM_1_ levels are almost always higher than the PM_2.5_ limit values both indoors and outdoors.

### 3.2. Comparison of PM Emission during Selected Smoking/Vaping Session

In Table 1 are reported the arithmetic mean (AM), with the respective standard deviation (SD), and the median, with the respective interquartile range (IQR), of outdoor PM_1_ levels found before and during each smoking/vaping session.

The results in Table 1 show an increase in outdoor PM_1_ levels during the smoking/vaping session compared to the levels measured before the related session for each device. The median outdoor PM_1_ levels increased from 44.0 to 57.5 for combustion products and from 23.0 to 34.0 for non-combustion products. PM_1_ levels significantly increase (*p*-value <0.05) for all the monitored devices except for IQOS^®^, which, although not statistically significant, caused a worsening of outdoor air quality. Looking at the AMs and SDs, the values are extremely variable during each smoking/vaping session.

Figure 4 reports the boxplots of outdoor PM_1_ levels for each device and graphically shows medians with respective IQRs during the smoking/vaping sessions.

RYO and JUUL^®^, respectively one traditional combustion product and a new heat-not-burn device, emitted the highest levels of PM.

Figure 5 shows for each considered product, the PM_1_ measurement (point by point) performed during each smoking/vaping session, highlighting the presence of peaks of PM_1_ levels in correspondence of the exhalation of the smoke.

Data reported in Figure 5 show an increase of PM_1_ levels of 93 and 190 times higher than the outdoor PM_1_ values before smoking session respectively for conventional cigarette and RYO. As well as considering the outdoor levels of PM_1_ emitted during the vaping of non-combustion products, we measured several peaks, of about 4, 34, 52 and 427 times higher, respectively, than the background PM_1_ values, for IQOS^®^, GLO^®^, JUUL^®^ and e-cig.

Figure 6 reports the indoor/outdoor ratios of PM_1_ levels for the environmental level and for smoking/vaping session of each device.

As shown in Figure 6, the indoor/outdoor ratios of PM_1_ levels during the smoking/vaping sessions of each device were reduced with respect to the ratio of the environmental level.

## 4. Discussion

The first relevant finding is related to the outdoor PM_1_ levels registered during the environmental measuring sessions. Indeed, the results demonstrated a worsening of outdoor air quality, during all the smoking/vaping sessions, especially when two or more products were used at the same time. Besides, the outdoor PM_1_ levels remain higher than the background level even when the cigarettes or the other products were extinguished (Figure 2 and Figure 3). These findings agree with the results of previous studies on outdoor air pollution due to cigarettes and possible exposure to passive smoking outdoors [12,34,35]. In particular, Repace et al. [34] measured the outdoor PM levels in proximity of a group of smokers (up to 10 people) outside the cafeteria entrance of an American university college, demonstrating that PM_2.5_ raised to 100-150 µg m^−3^/24h. Ruprecht et al. [12] compared the outdoor air quality by measuring PM levels, respectively, in a high-traffic area and a pedestrian area in which were located a high number of outdoor restaurants and bars, where people commonly smoke. Even though PM_1_ levels were similar in the two streets during morning hours, in the evening, PM_1_ levels measured in the pedestrian area were significantly higher (more than twice) with respect to those found in the high traffic street and correlated with the number of cigarettes smoked outdoors. All these results together with those obtained in the present study demonstrate that the common understanding that smoking outdoor is safe must be considered wrong as it leads to the possibility of passive smoke exposure for those close to smokers. In particular, it has been proved that people with respiratory diseases, such as asthma and chronic obstructive pulmonary disease (COPD), who are exposed to short-term SHS in outdoor areas, have a worsening in respiratory parameters [36]. It would be interesting to study the effects of outdoor long-term ETS exposure both in these subjects and in healthy non-smokers.

This consideration can be taken not only for conventional tobacco products, but also for non-combustion products. Indeed, even if the effect of conventional cigarettes on outdoor pollution is more relevant, the results of the environmental monitoring demonstrated a significant increase in outdoor PM_1_ levels both for combustion and non-combustion products. The comparison of the PM_1_ levels before and during the smoking/vaping session of each selected product (Table 1) confirm a worsening (almost always statistically significant) of outdoor air pollution when combustion and non-combustion products were used. There was only an exception found during the use of an IQOS^®^ (PM_1_ levels ranging from 39.25 [3.34] to 46.01 [24.09], p-value <0.181), that may be explained by the fact that e-cig aerosol is only produced during the activation of the device [37] and by specific smoking ways of each smoker. Indeed, we obtained extremely variable values during each smoking/vaping session (Figure 5), that can be due to the specific smoking way, but also to the specific characteristics of each device and the PM_1_ peaks determined by smoke exhalation during each puff. This is in line with results reported in our previous study on indoor PM contaminations during the indoor use of conventional cigarettes and electronic or heat-not-burn devices [17].

The demonstration of outdoor air pollution and possible ETS exposure determined by combustion and non-combustion products during their use outdoor is of particular importance for all the products. There is still little evidence of outdoor air pollution from smoked combustion products outdoors and, in our knowledge, this is the first study evaluating the outdoor air pollution generated by the outdoor use of non-combustion devices such as IQOS^®^, JUUL^®^ and GLO^®^. In contrast, these devices are very popular and commonly used worldwide; thus, it is essential to produce scientific evidence for both active and passive vapers. For example, JUUL^®^, one of the most recent electronic devices, was introduced in 2015 and it had captured more than 70% of the branded e-cigarette market in the United States [38], appealing in particular young people. Besides, Vallone et al. [39], found that in the United States JUUL^®^ use increased from 6.1% in 2018 to 13.5% in 2019 for those aged 15-34 years. It should be interesting to measure the SHS exposure of subjects standing near the smoker/s during the use of combustion and non-combustion products by the use of biological markers of exposure, such as urinary cotinine, a well-known indicators of active and passive exposure to smoke [40], urinary unmodified benzene [41], or other substances or their metabolites in biological matrices [42].

As regards to the environmental measurements performed indoor, the results evidence that indoor air quality worsens when combustion and non-combustion products were used outdoor, especially when used simultaneously. These results are in line with those from a previous study performed to evaluate indoor and outdoor ETS levels in some public places presenting indoor smoking bans in Barcelona. For this purpose, the authors measured PM_2.5_ levels in four locations of each building not potentially exposed to sources of PM_2.5_ other than tobacco smoke (indoor hall, outdoor main entrance, indoor control and outdoor control areas) and recorded statistically significant higher PM_2.5_ levels in the hall and the main entrances than in the control areas. A positive association between PM_2.5_ levels and airborne nicotine levels found in the same locations further confirmed that the source of PM_2.5_ was the smoke of tobacco products [12]. Similarly, another study was carried out to assess indoor and outdoor ETS levels by measuring PM_2.5_ levels in some indoor and outdoor areas of some hospitals of the Catalan Network for Smoke-Free Hospitals; the results demonstrated that the highest levels of PM_2.5_ were registered in outdoor areas, where smoking was allowed [32].

It is important to note that the number of outdoor particles that indoor environments receive is related to the particle infiltration factors, which is characteristic of each environment, to the outdoor aerosol levels and to the particles size distributions [43]. We elaborated the indoor/outdoor ratios for the PM_1_ levels measured before smoking/vaping session and during the use of each selected device. The results evidenced a reduction of the ratio in all cases respect to the environmental level and a very great variability of the ratio. This finding is in line with those reported by a recent review on this issue, reporting ratios of PM_10_ and PM_2.5_ levels widely different between and within indoor and outdoor environments. The indoor/outdoor ratios of PM levels recovered in the revised papers ranged from about the unit (gym, offices, classes, library) to 30 (air-conditioned classroom during cleaning hours in a rainy day [44]).

Another relevant finding of the present study is related to the comparison between our results and the WHO air quality guideline values for PM_2.5_ and PM_10_: indoor and outdoor PM_1_ levels are almost always higher than the WHO value for 24-h means PM_2.5_ levels (25 µg m^−3^). Even, outdoor PM_1_ levels exceeded the WHO values for 24-h means PM_10_ levels (50 µg m^−3^) during every smoking/vaping session.

The present study has some limitations. First of all, the study was performed measuring what happens in a real situation where some experimental conditions have not been checked. Indeed, we measured PM levels during the smoking sessions performed by real smokers, and we did not use smoking machine; thus, our results might be influenced by specific ways of smoking. However, the results are relevant because they demonstrated, with objective data, a worsening of both outdoor and indoor air quality when one or more smokers smoked/vaped outdoor. In addition, in our study we measured only the levels of PM and we did not evaluate other pollutants emitted during smoking or vaping. It would, therefore, be desirable to carry out additional experiments under controlled conditions, characterizing the chemical composition of PM and evaluating other substances of the released aerosol that can contaminate indoor and outdoor air.

## 5. Conclusions

All the results presented above highlight two important considerations: firstly, smoking/vaping outdoors causes a relevant increase in PM_1_ levels in the proximity of the smoker/s determining the possibility of ETS exposure for those who are near the smoker/s, also outdoors. Secondly, smoking/vaping outdoor, but in the proximity of an entrance of a building, causes an increase in indoor PM_1_ levels, too; this finding means that indoor environments with smoking bans are not entirely free from smoking coming from outside. Thus, these results imply the need for a revision of the smoke-free laws especially for outdoor areas. These laws should also include electronic devices and heat-not-burn products as they determine a significant worsening of outdoor air quality during their use. Indeed, some laws on outdoor smoking bans have already been enacted, but considering outdoor smoking under this relatively new perspective, they should be extended. Thus, it is essential to raise society awareness of the dangers of smoking outdoors by implementing health promotion interventions for outdoor smoking, both for combustion and non-combustion products. Outdoor smoking does not guarantee the safety of non-smokers who are nearby and, therefore, smoking bans should be extended to all outdoor areas of public interest.

## Figures and Tables

**Figure 1:** Monitored area.

**Figure 2:** Levels of PM_1_ (μg m^−3^), expressed in Log(10)PM_1_, measured, respectively, outdoors (**a, b**) and indoors (**c, d**) during the afternoon measuring session. **1.** cig = one conventional cigarette; RYO = “Rolled your own” hand-rolled cigarette; e-cig = electronic cigarette. Red dropped line: WHO guideline value for PM_2.5_ (24-h mean). Blue dropped line: WHO guideline value for PM_10_ (24-h mean).

**Figure 3:** Levels of PM_1_ (μg m^−3^), expressed in Log_(10)_PM_1_, measured, respectively, outdoors (**a, b, c**) and indoors (**d, e, f**) during the morning measuring session. **1.** cig = one conventional cigarette; RYO = “Rolled your own” hand-rolled cigarette; e-cig = electronic cigarette. Red dropped line: WHO guideline value for PM_2.5_ (24-h mean). Blue dropped line: WHO guideline value for PM_10_ (24-h mean).

**Figure 4:** Boxplots of outdoor PM_1_ levels (μg m^−3^) for each device. * 1 cig = one conventional cigarette; RYO = “Rolled your own” hand-rolled cigarette; e-cig = electronic cigarette.

**Figure 5:** Outdoor PM_1_ levels (expressed in Log_(10)_PM_1_), measured point by point, for each device during a smoking/vaping session. Red dropped lines represent the arithmetic mean of outdoor Log_(10)_PM_1_, before starting smoking each device. * 1 cig = one conventional cigarette; RYO = “Rolled your own” hand-rolled cigarette; e-cig = electronic cigarette.

**Figure 6:** Indoor/outdoor ratios of PM_1_ levels for environmental level and during the smoking/vaping sessions of each device. * 1 cig = one conventional cigarette; RYO = “Rolled your own” hand-rolled cigarette; e-cig = electronic cigarette.

**Table 1:** Outdoor PM_1_ levels (μg m^−3^) for each device, before and during each smoking/vaping session.

Type of Smoke Product	Before Smoking/Vaping Session		During Smoking/Vaping Session		*p*-Value
	AM [SD] ^1^	Median [IQR] ^2^	AM [SD] ^1^	Median [IQR] ^2^	
**1 cig** *	18.10 [1.58]	18.00 [2.00]	106.84 [214.07]	44.00 [58.00]	<0.001
**RYO** *	25.10 [1.04]	25.00 [2.00]	221.61 [665.99]	57.50 [93.00]	<0.001
**e-cig** *	28.81 [1.94]	23.00 [2.00]	394.82 [1317.66]	23.00 [29.00]	<0.023
**IQOS^®^**	39.25 [3.34]	39.00 [4.00]	46.01 [24.09]	41.00 [9.00]	<0.181
**GLO^®^**	35.85 [1.09]	36.00 [2.00]	106.30 [191.92]	43.00 [24.00]	<0.001
**JUUL^®^**	29.25 [1.59]	29.00 [2.00]	159.13 [304.74]	34.00 [107.00]	0.003

^1^ AM = Arithmetic mean, SD = Standard deviation; ^2^ IQR = Interquartile range. * 1 cig = one conventional cigarette; RYO = “Rolled your own” hand-rolled cigarette; e-cig = electronic cigarette.

## Appendix A

The Smoke-free Department Working Group
Susanna Caminada—Sapienza University of Rome
Barbara Dorelli—Sapienza University of Rome
Monica Giffi—Sapienza University of Rome
Matteo Iachini—Sapienza University of Rome
Federica Anna Pirro—Sapienza University of Rome
Roberta Noemi Pocino—Sapienza University of Rome
Matteo Ricciardi—Sapienza University of Rome
Filippo Sandorfi—Alma Mater Studiorum–University of Bologna
Alessandro Sindoni—Sapienza University of Rome
